The article "Evaluation of PAX8 expression promotes the proliferation of stomach Cancer cells" was retracted in 2021. Reason: duplicate publication.

# Evaluation of PAX8 expression promotes the proliferation of stomach Cancer cells

**DOI:** 10.1186/s12860-019-0245-9

**Published:** 2019-12-27

**Authors:** Liang-Yu Bie, Ning Li, Wen-Ying Deng, Xiao-Yu Lu, Ping Guo, Su-Xia Luo

**Affiliations:** 1 Department of Oncology, Affiliated Cancer Hospital of Zhengzhou University Henan Cancer Hospital, Zhengzhou, NO. 127, Dongming Road, Jinshui District, Zhengzhou, 450008 Henan China; 2 Department of Pathology, Affiliated Cancer Hospital of Zhengzhou University Henan Cancer Hospital, Zhengzhou, 450008 Henan China; 3 Department of Oncology, the First Affiliated Hospital of Nanyang Medical College, Nanyang, 473061 Henan China

**Keywords:** PAX8, Expression, Proliferation, Stomach Cancer

## Abstract

**Background:**

PAX8 was not only a mitotic factor, but identified as a transcription factor involved in the prognosis of human tumor patients. Elucidating the function of PAX8 on the pathology of stomach cancer was meaningful.

**Results:**

PAX8 was found to be upregulated in primary stomach cancer tissue and the TCGA stomach cancer dataset. Interestingly, SOX13 and PAX8 showed consistent expression patterns, and the combined high PAX8 and SOX18 expression induced a worse prognosis of stomach cancer patients. SOX13 was further identified as a transcription factor of PAX8, and further affect Aurora B and Cyclin B1 expression, two cell cycle related factors of the downstream of PAX8, including. Furthermore, PAX8 depletion inducted G1-phase arrest and the decrease of EdU incorporation, cell viability and colony formation can be rescued by SOX13 overexpression.

**Conclusions:**

SOX13 participated in the elevated expression of PAX8, which promote the proliferation of stomach cancer cells. Therefore, SOX13 mediated PAX8 expression was recognized as a tumor-promoting role in stomach cancer.

## Background

Stomach cancer was one of the high risk of cancer-related deaths worldwidely, with the characteristic of rapid pathological progress and low screening efficiency [1, 2]. Recently, stomach cancer patients undergoing traditional treatment, including surgery, chemotherapy and other therapies, showed high recurrence, causing widespread concern [3–5]. However, drugs targeting to cell proliferation regulator, which were developed for the suppression the tumor malignant proliferation, have shown a strong anti-cancer effect and significantly reduced the risk of death and recurrence of patients, binging new light to the treatment of stomach cancer [6, 7]. Therefore, the study of the molecular mechanism of the malignant proliferation of stomach cancer cells is of great significance for exploring potential therapeutic targets and the development of drugs for stomach cancer [8].

Transcription factor PAX8, an important regulator of embryo development [9], was associated with abnormal kidney development in male PAX8 knockdown mice and endometrial dysfunction in female PAX8 knockout mice [10]. Notably, PAX8 was highly expressed in human malignancies, and significantly enhanced the proliferation of tumor cells via regulating the expression of cell cycle regulator, such as Aurora B and Cyclin B1 [11, 12]. Upregulation of PAX8 in endometrial and ovarian cancer tissues [13, 14] was accompanied with a higher risk of death and high recurrence in patients [15]. However, the clinical significance of PAX8 and its function on proliferation of human stomach cancer was confusing.

In addition to maintain the stemness of stem cell by involved in regulating the Wnt / β-catenin signaling pathway, SOX13 has also been reported to be abnormally expressed in cancer tissues containing poorly differentiated cells [16, 17]. SOX13 containing the HMG-box domain can provide a platform for recruiting other transcriptional molecules to regulate the transcription of target genes by combining HMG-box homologous sequences in the promoter region of target genes [18, 19]. SOX13 has been reported as a molecular marker for the diagnosis of potential malignant tumors, and its high expression in malignant tumors usually resulted with a poor survival prognosis for patients [20]. However, the expression pattern and molecular function of SOX13 in stomach cancer was rarely studied.

In our study, the clinical significance and molecular function of SOX13 and PAX8 in stomach cancer were discussed, and the proliferation of stomach cancer cells promoted by SOX13-regulated PAX8 expression was expounded, providing a new insight into the mechanism of malignant proliferation of stomach cancer cells.

## Result

### PAX8 and SOX13 are upregulated in stomach cancer

The TCGA stomach cancer database was first used to retrieve the expression patterns of all the PAX family transcription factors, and the expression of PAX8 was found to be significantly up-regulated in stomach cancer tissues compared to normal tissues (Fig. 1a). Although the cancer-promoting role of PAX8 in most types of tumors has been widely reported, the clinical significance and molecular function of PAX8 in stomach cancer remain puzzling. In order to verify whether PAX8 is related to the pathological progression of stomach cancer, the expression pattern of PAX8 in stomach cancer tissues with different pathological progression was further explored. Interestingly, in four stomach cancer tissues with different stages, the expression of PAX8 showed an increasing trend by the pathological stages (Fig. 1b).

**Fig. 1:** Expression pattern of PAX8 and SOX13 in stomach cancer. **(a)** Expression lever of PAX8 in stomach cancer contract to normal tissues based on TCGA dataset. **(b)** PAX8 mRNA expression lever in four different grades of cancer samples based on TCGA dataset. **(c)** SOX13 co-expressed with PAX8 in stomach cancer based on TCGA dataset. **(d, e)** PAX8(**d**) and SOX13(**e**) mRNA expression pattern in 36 pairs of human stomach cancer tissues (Cancer) and adjacent tissues (Normal). **(f)** SOX13 co-expressed with PAX8 in 36 human stomach cancer tissues. **(g, h)** Relative mRNA and protein expression level of PAX8 and SOX13 in four stomach cancer cell lines compared to GES1 cells. GAPDH served as endogenous control

To further explain the up-regulated expression of PAX8 mRNA in stomach cancer, we were interested in the fact that HMG-box transcription elements were found to be widely present in the promoter region of PAX8, suggesting that the increased expression of PAX8 mRNA might be related to HMG-box contained transcription factors. By analyzing the TCGA stomach cancer database, we found that the expression of HMG-box domain contained SOX13 was also up-regulated, and the SOX13 expression was positively correlated with the expression pattern of PAX8 (r = 0.6567, *p* < 0.001) (Fig. 1c).

Furthermore, qRT-PCR assay revealed that SOX13 showed consistent up-regulated expression patterns as similar as PAX8 in 36 pairs of stomach cancer tissues (Fig. 1d, e). In addition, spearman correlation analysis of the mRNA lever of PAX8 and SOX13 in stomach tumor tissues suggested a strong positive correlation (r = 0.6567, *p* < 0.001), consistent with TCGA-based results (Fig. 1f).

To explore the differences of PAX8 and SOX13 expression pattern in different stomach cancer cell lines, SOX13 was found to significantly up-regulated in stomach cancer cell lines as the expression pattern of PAX8, especially in MGC803 and AGS cell lines, by comparing PAX8 and SOX13 expressed in 4 stomach cancer cell lines with GES1 cells (Fig. 1g, h). However, it was noted that the mRNA and protein level of PAX8 was overexpressed in cell lines where SOX13 mRNA and protein were also significantly up-regulated, suggesting the positive correlation of SOX13 and PAX8 (Fig. 1g, h).

### Upregulated SOX13 and PAX8 was associated with worse prognosis of stomach cancer patients

Immuno-histochemical staining of stomach cancer specimens was performed to explore the distribution of PAX8 and SOX13 in stomach cancer tissues. The staining section indicated that PAX8 were mainly distributed in the nucleus, as the stain result of SOX13 (Fig. 2a). Furthermore, 36 clinical tissues were classified according to the staining levels of PAX8 and SOX13, and the results indicated that the protein of SOX13 and PAX8 expressed in tissues were significantly different (χ2 test, *p* = 0.0361). In brief, 47.22% (17/36) of stomach cancer patients was accompanied with SOX13 and PAX8 overexpression, while only 22.22% (8/36) of patients showed a lower expression of PAX8 and SOX13 (Fig. 2b), indicating the probability that PAX8 shared the same expression pattern as SOX13 in stomach cancer.

**Fig. 2:** Combined PAX8 and SOX13 expression may predict the overall survival in patients with stomach cancer. **(a)** Immuno-histochemical analysis of PAX8 and SOX13 expression in 36 stomach cancer samples. **(b)** Correlation of PAX8 and SOX13 was statistically analyzed. **(c, d)** Overall survival of patients with stomach cancer was calculated using Kaplan–Meier analysis according to low and high PAX8**(c)** or SOX13**(d)** staining. The *P* values were calculated by log-rank test. **(e)** Overall survival of patients with stomach cancer was calculated according to combined PAX8 and SOX13 staining level

Furthermore, weather the level of SOX13 and PAX8 in stomach cancer was correlated with the survival of patients was explored, in order to clarify the clinical significance of SOX13 and PAX8. By comparing the survival curves, it was found that not patients with high level of PAX8 significantly resulted with worse survival compared to patients with low PAX8 expression, but also SOX13 did (Fig. 2c, d). In stomach cancer patients with the same expression patterns of SOX13 and PAX8, combined low SOX13 and PAX8 expression was found to result with a better overall survival rate, but not up-regulated SOX13 and PAX8 (Fig. 2e). These results suggest the clinical significance of SOX13 and PAX8 in stomach tumors, which can be used as potential biological indicators for the survival of patients with stomach cancer.

### SOX13 regulates the transcription of PAX8 in stomach cancer

In order to verify that the up-regulated expression of PAX8 in stomach cancer is related to SOX13, we verified whether SOX13 can regulate PAX8 expression in stomach cancer cell lines. It was first found that different amounts of SOX13 overexpression could cause the associated increase of PAX8 mRNA and protein expression level in AGS and MGC803 cells (Fig. 3 a, b). Moreover, silencing SOX13 can down-regulate PAX8 mRNA and protein expressed in AGS and MGC803 cell lines, while SOX13 overexpression can rescue the down-regulation of PAX8 to some extent caused by SOX13 knockdown. However, even overexpressed SOX13 mutants (SOX13 ins6), in which six amino acids were inserted into the HMG-box of SOX13 to deprive its ability to bind with the HMG-box DNA sequence, cannot reverse the decline in PAX8 expression (Fig. 3c, d). These results confirmed that SOX13 was one of the factors regulating PAX8 expression in stomach cancer.

**Fig. 3:** PAX8 expression pattern can be regulated by SOX13 in stomach cancer. **(a, b)** Relative mRNA and protein expression of PAX8 in SOX13 overexpressed AGS and MGC803cell lines. **(c, d)** SOX13 can rescue mRNA and protein expression level of PAX8 in AGS and MGC803 cell lines. **(e)** PAX8 promoter deletions fused to the luciferase reporter gene were transfected with SOX13 in AGS cells. **(f)** ChIP assay was used to examine the interaction of PAX8 promoter with SOX13 in AGS and MGC803 cell lines. **(g)** SOX13 mediated PAX8 targeted genes expression in AGS and MGC803 cell lines

Since SOX13 has been proved to regulate the expression of PAX8 in stomach cancer, luciferase assay was further used to explore the combination of SOX13 with the promoter region of PAX8, in order to verify that SOX13 was a transcription factor of PAX8. Although SOX13 overexpression was found to significantly increase the expression of reporter genes containing the PAX8 promoter, SOX13 lost its ability to promote reporter gene expression, when the PAX8 promoter region was reduced by more than 600 bp on the far terminal (Fig. 3e), suggesting that SOX13 may bind with the − 300~ − 600 bp regions of the PAX8 promoter to regulate PAX8 expression. Furthermore, ChIP-qRCR assay showed that SOX13 could significantly enrich the − 300~ − 600 bp region of PAX8 promoter, confirming the interaction between SOX13 and PAX8 promoter (Fig. 3f).

Previous studies have shown that Aurora B and Cyclin B1, as mitotic regulators, can be regulated by PAX8 and thus affect the progression of tumor cell cycle, which promoted us to speculate whether SOX13-regulated PAX8 expression can affect the expression of Aurora B and Cyclin B1 in stomach cancer. PAX8 silencing can significantly cause the silencing of Aurora B and Cyclin B1, the expression of Aurora B and Cyclin B1 were recovered, when PAX8 was expressed in AGS and MGC803 cells, confirming that PAX8 can regulate the expression of Aurora B and Cyclin B1 in stomach cancer (Fig. 3g). Moreover, wild type SOX13 expression also restores the mRNA level of Aurora B and Cyclin B1, in parallel with the upregulated expression of PAX8 to a certain extent (Fig. 3g), suggesting the notion that SOX13-regulated PAX8 expression affects the expression pattern of Aurora B and Cyclin B1 in stomach cancer.

### SOX13-mediated PAX8 expression promotes cellular proliferation in stomach cancer

In view of the positive effect of SOX13-regulated PAX8 expression on cellular Aurora B and Cyclin B1 expression, SOX13-regulated PAX8 expression function on cell cycle was detected. And flow cytometry assay showed that PAX8 knockdown induced G1-phase arrest in AGS and MGC803 cell lines, which could be rescued by SOX13 overexpression (Fig. 4 a, b). What’s more, the overexpression of SOX13 can significantly increase the decline of EdU positive cells induced by PAX8 knockdown, no matter in AGS cells or in MGC803 cells, indicating that SOX13-mediated PAX8 expression can promote the progression of cell cycle in stomach cancer (Fig. 4 c, d).

**Fig. 4:** SOX13 dependent PAX8 expression promotes cell proliferation in stomach cancer. **(a, b)** Flow cytometry analysis of cell cycle distribution in PAX8 silenced AGS and MGC803 cell lines and controls. **(c, d)** EdU incorporation assay showed the percentage of in S-phase in PAX8 silenced AGS and MGC803cells. **(e)** CCK8 assay showed cells viability in PAX8 silenced AGS and MGC803 cells. **(f, g)** The clone formation assay in PAX8 silenced AGS and MGC803 cells and controls

Next, whether PAX8 function on the cellular viability in stomach cancer was detected, which was one of the indicators for malignant proliferation of tumor cells. The results showed that PAX8 knockdown could directly weaken the viability of stomach cancer cells, while the up-regulation of PAX8 expression induced by SOX13 overexpression restored the cell viability (Fig. 4 e). Consistently, SOX13 overexpression can significantly increase the PAX8 silencing-induced decrease of clone formation in both AGS cells and MGC803 cells, indicating that SOX13-mediated PAX8 can promote the tumorigenicity of stomach cancer cells (Fig. 4 f, g). Therefore, the expression of PAX8 regulated by SOX13 can promote the progress of stomach cancer cell cycle, showing the capbilty to promote tumorigenicity of stomach cancer cells.

## Discussion

Exploring for the feasible targets to inhibit malignant tumor cell proliferation has become one of the direction of development of new cures for cancer, including cancers of the stomach, except for the traditional treatment for stomach cancer [21, 22]. Therefore, it is still a hot topic in the research of stomach cancer to find the molecular and signal transduction pathways related to proliferation regulation [23, 24]. Studies have shown that up-regulated expression of PAX8 in malignant tumors, including digestive and urinary tumors, has also been shown to be a biomarker for the diagnosis of ovarian and kidney cancer, and has been the focus of researchers [25, 26]. Recently, the effect of PAX8 has been indicated to support the clearance of tumor cells and be the prediction of survival time in tumor patients [12]. The proliferation of rat thyroid cells can be significantly inhibited by silencing the expression of PAX8, revealing the importance of PAX8 in regulating the proliferation of thyroid cells [27]. In addition, the high expression of PAX8 has been shown to regulate the lifespan of tumor cells by activating telomerase activity in gastrointestinal and nervous system tumors [28]. Although these studies have revealed PAX8 function on the cell cycle progression in different types of tumors, the effect of PAX8 on the cellular proliferation in stomach cancer has not been reported.

In this study, we identified that PAX8 was highly expressed in stomach cancer, and that the worse prognosis was found in stomach cancer patients with high PAX8 expression. Furthermore, PAX8 had the ability to regulate the expression of Aurora B and Cyclin B1 in stomach cancer cells, which further revealed the capability of PAX8 to affect the cellular tumorigenicity in stomach cancer by regulating the progression of stomach cancer cell cycle. In addition, the downregulation of PAX8 can indeed arrest the cell cycle in stomach cancer and reduce the tumorigenesis of stomach cancer cells, indicating that PAX8 played a carcinogenic role in the pathological development of stomach cancer. Whatever, these results suggest the potential value of PAX8-related signaling pathways in the diagnosis and treatment of stomach cancer.

Members of the SOX family expressed in embryonic tissue or stem cells have the ability to maintain cellular stemness and regulate differentiation [29, 30]. In recent years, HOM-box domain contained SOX family transcription factors have been found to be abnormally expressed in tumor cells and involved in regulating tumor cell growth, such as SOX10 and SOX12 [31]. SOX10 can be used as a serum biomarker to increase the efficacy of GPM6B and COL9A3 in the diagnosis of basal breast cancer and the prognosis of patients, which was mainly related to its function on the proliferation of breast tumor cell [31]. Similarly, the upregulation of SOX12 was aslo indentified as a biomarker of poor prognosis in colon cancer patients [32]. In addition, the proliferation of colon cancer cells was significantly inhibited by knocking down SOX12 expression [33], suggesting the significance of SOX family in regulating the proliferation of cancer cells. In this study, the up-regulated expression of SOX13 was found to be positively correlated with the expression of PAX8 in stomach cancer tissues. Interestingly, SOX13 was confirmed as a transcription factor of PAX8 to regulate the expression of PAX8 and its downstream cycle-related Aurora B and Cyclin B1 in stomach cancer cells, which promoted the progression of stomach cancer cell cycle and enhanced the tumorigenicity of stomach cancer cells, suggesting that SOX13, as one of the tumor cell cycle regulators, was oncogene in stomach cancer.

## Conclusions

In conclusion, PAX8 were confirmed to be overexpressed in primary stomach cancer, and SOX13 mediated PAX8 expression promoted the proliferation and tumorigenesis of stomach cancer cells. Furthermore, up-regulated SXO13 and PAX8 showed an unfavorable factor for the clinical prognosis of patients. However, for exploring the mechanism of cancer cellular proliferation, it will be significant to further explore the network of PAX8 in stomach cancer.

## Methods

### Cell lines

Stomach cancer cell lines (MKN45, MKN28, MGC803, AGS) and GES1 cell lines were purchased from American Type Culture Collection (ATCC, USA). MKN45, MKN28, MGC803 and AGS were cultured in RPM1636 Medium containing 10% fetal bovine serum (Gibco) and GES1 in Dulbecco’s Modified Eagle Medium (DMEM) containing 15% fetal bovine serum (Gibco).

### Human tissue specimens

The stomach cancer tissues and para-cancer tissues of 36 cases were collected from stomach cancer patients in Henan Cancer Hospital. All patients signed the informed consent and did not receive chemotherapy or radiotherapy before surgery. Some of the tissue was used for gene expression analysis, while the rest was fixed with formalin for immune-histochemical analysis. All patients were collected and kept complete medical records. The experiment was supported by the institute’s ethics committee.

### Immunohistochemistry

Formalin solution immobilized tissues were dewaxed in xylene solution and ethanol solution. Endogenous peroxidase was quenched with 1% H2O2 solution. The specimens were rinsed in PBS and sealed with 3% BSA at room temperaturefor 1 h. Protein expression in tissues was detected with SOX13 and PAX8 primary antibody (Abcam) and DAB labeled secondary antibodies. The staining results were analyzed by Image J software.

### Virus packaging and infection

Lentiviruses containing the shRNA targeting SOX13 or PAX8 were generated following the protocol described by Addgene. The plasmids were co-transfected into the packaged cell line HEK293T. After 48 h, the virus supernatant was collected, filtered and clarified, and concentrated by super-centrifugation. 5 × 10^5^ AGS and MGC803 cells (30–40% fused) placed in a 60 mm dish were infected with a concentrated virus and 5 μg/ml of polybrene. 24 h later, cells were screened with 2 μg/ml of proteromycin (Sigma) for 1 week.

### RNA extraction and qRT-PCR

Total RNA was isolated from tissues or cells using Trizol reagent (Invitrogen). The first strand of cDNA was obtained using RNA as template with reverse transcription kits (TOYOBO). Quantitative analysis of all gene transcripts was performed with the Power SYBR Green PCR Master Mix (TOYOBO) on the ABI 7500 series system (Applied Biosystems, Foster City, CA). The internal reference gene was GAPDH, and the primers are listed in Table 1.

**Table 1:** Primers used for quantitative real-time PCR

Gene	Primers (5′ to 3′, forward/reverse)
*SOX13*	CCAGAGGGTAATGGGTCCC / TGGCTTCCATAGAGTTCCTTCC
*PAX8*	ATCCGGCCTGGAGTGATAGG / TGGCGTTTGTAGTCCCCAATC
*Aurora B*	CAGAAGAGCTGCACATTTGACG / CCTTGAGCCCTAAGAGCAGATTT
*Cyclin B1*	ACGAAGGTCTGCGCGTGTT / CCGCTGGCCATGAACTACCT
*GAPDH*	GGAGCGAGATCCCTCCAAAAT / GGCTGTTGTCATACTTCTCATGG
*PAX8 promote*	GAACAGAGGGAATGGCTTC/CCAGAAGTGAGAGGGATGGT

### Chromatin immunoprecipitation (ChIP assay)

ChIP assay was performed with EZ-ChIP Kits (Millipore) to verify SOX13 local on the PAX8 promoter region according to kit instructions. Immunoprecipitation was performed with SOX13 antibody (Abcam) to obtain targeted DNA fragments. Quantitative PCR analysis was performed with the Power SYBR Green PCR Master Mix on the ABI 7500 sequence detection system (Applied Biosystems, Foster City, CA).

### Luciferase assay

AGS cells were transfected with pGL3 report vectors with different PAX8 promoter fragments with plasmids expressing SOX13. Renilla vector was used as a negative control. Cells were collected 36 h later and luciferase activity was measured with the Double Luciferase Reporter Assay System (Promega). Firefly luciferase activity were normalized to Renilla luciferase activity.

### Flow cytometry

Trypsin collected cells were washed with PBS and fixed overnight at − 20 °C with 70% ethanol. After centrifugation, the fixed cells were washed with PBS and stained for 20 min with 100 μg/ml RNase A (Sigma) and 50 mg/ml propidium iodide (Sigma) in 500 μl PBS. Cell cycle data were acquired by FACSCalibur system (BD Biosciences).

### EdU incorporation assay

About 2000 cells of different genotypes were planted on 96-well plates and cultured at 37 °C for 24 h. After that, 20 mM EdU was added and continued to be cultured for 2 h. Cells were collected, fixed with 4% formaldehyde, stained with EdU Apollo@594 in vitro imaging kit (Ribo) according to the instructions. EdU incorporation rate was determined by leica inverted fluorescence microscopy.

### Colony formation

One thousand cells of different genotypes were plated in three copies in a 6-well dish. After 14 days of training, the colonies were dyed with 0.5% crystal violet /20% ethanol and counted. Results were normalized to plating efficiencies. Results are expressed as the average of three independent experimental data.

### Statistical analysis

All experiments were independently repeated for 3 times, and results were expressed as mean ± SD. GraphPad Prism software (version 5.01) was used for statistical analysis, and *p* < 0.05 was considered statistically significant (* p < 0.05, ** *p* < 0.01, *** *p* < 0.001). The paired t-test was used to analyze the gene expression differences in the paired tissues, and the double-tailed *t*-test was used to evaluate the other two groups of independent repeated experiments. The distribution differences of SOX13 and PAX8 in tissues were analyzed by χ^2^ test.

## Data Availability

All data generated or analysed during this study are included in this published article or supplementary files.

## Abbreviations

CCK8: Cell count kit-8
Edu: 5-Ethynyl-2′- deoxyuridine
PAX8: Paired box 8
qRT-PCR: Quantitative reverse transcribe-polymerase chain reaction
SOX13: SRY-Box 13
